The article "IoMT-Based Mitochondrial and Multifactorial Genetic Inheritance Disorder Prediction Using Machine Learning" was published in 2022. Journal: Comput Intell Neurosci.

# IoMT-Based Mitochondrial and Multifactorial Genetic Inheritance Disorder Prediction Using Machine Learning

**DOI:** 10.1155/2022/2650742

**Published:** 2022-07-21

**Authors:** Atta-ur Rahman, Muhammad Umar Nasir, Mohammed Gollapalli, Suleiman Ali Alsaif, Ahmad S. Almadhor, Shahid Mehmood, Muhammad Adnan Khan, Amir Mosavi

**Affiliations:** ^1^Department of Computer Science (CS), College of Computer Science and Information Technology (CCSIT), Imam Abdulrahman Bin Faisal University, P.O. Box 1982, Dammam 31441, Saudi Arabia; ^2^Riphah School of Computing and Innovation, Faculty of Computing, Riphah International University, Lahore Campus, Lahore 54000, Pakistan; ^3^Department of Computer Information Systems (CIS), College of Computer Science and Information Technology (CCSIT), Imam Abdulrahman Bin Faisal University, P.O. Box 1982, Dammam 31441, Saudi Arabia; ^4^Department of Computer, Deanship of Preparatory Year and Supporting Studies, Imam Abdulrahman Bin Faisal University, P.O. Box 1982, Dammam 31441, Saudi Arabia; ^5^College of Computer and Information Sciences (CCIS), Jouf University, Saudi Arabia; ^6^Department of Software, Gachon University, Seongnam 13120, Republic of Korea; ^7^John von Neumann Faculty of Informatics, Obuda University, Budapest 1034, Hungary; ^8^Institute of Information Engineering, Automation and Mathematics, The Slovak University of Technology in Bratislava, Bratislava 81107, Slovakia; ^9^Faculty of Civil Engineering, TU-Dresden, Dresden 01062, Germany

## Abstract

A genetic disorder is a serious disease that affects a large number of individuals around the world. There are various types of genetic illnesses, however, we focus on mitochondrial and multifactorial genetic disorders for prediction. Genetic illness is caused by a number of factors, including a defective maternal or paternal gene, excessive abortions, a lack of blood cells, and low white blood cell count. For premature or teenage life development, early detection of genetic diseases is crucial. Although it is difficult to forecast genetic disorders ahead of time, this prediction is very critical since a person's life progress depends on it. Machine learning algorithms are used to diagnose genetic disorders with high accuracy utilizing datasets collected and constructed from a large number of patient medical reports. A lot of studies have been conducted recently employing genome sequencing for illness detection, but fewer studies have been presented using patient medical history. The accuracy of existing studies that use a patient's history is restricted. The internet of medical things (IoMT) based proposed model for genetic disease prediction in this article uses two separate machine learning algorithms: support vector machine (SVM) and K-Nearest Neighbor (KNN). Experimental results show that SVM has outperformed the KNN and existing prediction methods in terms of accuracy. SVM achieved an accuracy of 94.99% and 86.6% for training and testing, respectively.

## 1. Introduction

Genes are the building blocks of heredity. They are passed down through the generations. They contain deoxyribonucleic acid (DNA), which includes protein-making instructions. A mutation is a change in one or more genes that happens on a regular basis. The mutation changes the gene's instructions for making a protein, leading it to either not work properly or not exist at all. This can lead to a genetic disorder, which is a serious illness. One or both parents can pass on a genetic mutation to their children. Everybody is susceptible to mutation at some point in their lives [1]. There are illnesses caused by mutations inherited from the parents at birth. Congenital mutations in a gene or a combination of genes that appear at different times in life might cause other disorders. A mutation of this type may occur at random or as a result of environmental factors [2].

### 1.1. Multifactor Genetic Disorder

These disorders are caused by mutations in numerous genes, and they are typically the consequence of a complex interplay of environmental and nutritional factors. It is sometimes referred to as a complicated or polygenic disease [3]. Cancer, diabetes, and Alzheimer's disease can all be linked to a multifactor genetic condition.

### 1.2. Mitochondrial Genetic Disorder

It is associated with mutations in the mitochondrial nonnuclear DNA. Each mitochondrial genome contains 5 to 10 circular DNA segments. During fertilization, they maintain their organelles as eggs. As a result, this condition is always inherited from the mother [3]. The mitochondrial genetic condition causes mitochondrial encephalopathy, lactic acidosis, stroke-like events, and eye damage. “Every year, about 140 million toddlers are born throughout the world, with ten million of these toddlers being born with a severe birth defect of genetic or partially genetic origin, many of which are identified late,” said Linguraru.

The genetic disease prediction challenge was first handled as a two-class classification issue for machine learning research, with a classification model consisting of true and false training data. Decision trees, K-NN, naïve Bayesian classifier, and binary SVM classifier were employed [4]. Positive training samples in binary classification systems contain genes associated with known illnesses, whereas negative samples do not. Machine learning technology may be used to detect the presence of a genetic condition utilizing a facial photograph taken at a point of care, such as a pediatric office, maternity ward, or general practitioner clinic, as well as the 'patient's medical history [5].

The major contributions of this study are given below:

- Proposed a IoMT-based machine learning model to predict mitochondrial and multifactorial genetic disorders.
- The proposed model will improve previously used machine learning techniques with the help of different simulation parameters.
- Proposed framework uses unique data preprocessing techniques to enhance the prediction results.
- The proposed model uses various statistical matrixes to check the performance and reliability.

## 2. Literature Review

The identification of the most likely disease candidate genes is an important issue in biomedical research, and several methodologies have been proposed [6, 7]. Formalized paraphrase Most early techniques, such as ToppGene [8], highlighted candidate genes by rating them according to morphological or behavioral systems and correlating these ranks to commonly identified illness genes. These schema techniques have the limitation of being unable to find indirect relationships between genes that do not yet share comparable characteristics or activities. Biological network-driven gene prioritizing approaches have recently been developed to solve this issue [6, 9–12].

The coverage of functional genomic data, where new high technologies have provided a huge quantity of behavioral data among biological components, has resulted in the development of such network-based approaches over application techniques as well as protein structures. Machine learning algorithms have recently been effectively implemented to many important biomedical problems [13, 14], including genetic code explanation [15], genetic analysis categorization [16, 17], deductive reasoning of gene monitoring networks [18], drug target prognosis [19, 20], and revelation of epigenetic interactions in malady statistics [21, 22], as well as pharmacology [23]. Machine learning has been used to predict disease-associated genes [24, 25]. The challenge is typically framed as a classification job in which known genetic disorders and biological data linked with medical history data are used to build a classification model that is then used to predict emerging genetic illnesses. So, more pragmatic techniques have been developed. In fact, unary classifiers that can only be trained from positive data have been proposed [26]. To combine data from various sources, this research employed a binary support vector machine. Because the remaining collection may contain genes for unknown disorders, semisupervised learning approaches such as semisupervised binary learning techniques [27] and positive and negative [28] were proposed. In previous research, they used machine learning for genome disorder prediction with the help of DNA sequencing data and unary classification. Due to sequencing data results, they are impactful but not efficient to predict different kinds of genetic disorders with perfect accuracy and on time. The major drawback in previous research is DNA sequencing data. Due to this, results vary from paternal to maternal genes and ignore most of the parameters like abortion counts, etc. The authors [29] employed fine Gaussian SVM on hepatitis C patients using public data and achieved 97.9% resultant accuracy. A previous study [30] used the IoMT architecture empowered with a deep neural network for intrusion detection and achieved a 15% increased test results.

In this research, we used different supervised machine learning approaches with the help of patient medical history to predict mitochondrial and multifactorial genetic inheritance disorders. With the help of this study, the proposed model easily overcomes the drawbacks of DNA sequencing and achieved the best prediction accuracy.  Table 1 shows the limitations of previous studies. It shows that Asif et al. [31] achieved 79% prediction accuracy empowered with RF and SVM used miRNA feature base dataset and having handcrafted features and imbalance data limitation. Alshamlan et al. [32] achieved 81% prediction accuracy empowered with the GBC algorithm used the SRBCT feature base dataset and having handcrafted features and imbalance gene sequence data limitation. KhaderKhader et al. [33] achieved 80.5% prediction accuracy empowered with BA and SVM used gene seq feature base dataset and having imbalance gene sequence limitation.

## 3. Materials and Methods

The ability to forecast genetic disorders allows doctors to provide drugs that are helpful to the patient's health, and patients may easily maintain their health before any severe complications arise. We employed machine learning techniques such as SVM and KNN to predict mitochondrial and multifactorial inheritance gene disease in this research. Following the prediction analysis, we highlighted the model with the best accuracy in this study.  Figure 1 shows our workflow from dataset selection to prediction.

The proposed model uses IoMT technology to gather data from numerous hospitals with the help of different digital devices which can vary from hospital to hospital. With the help of IoMT, the collection of process data is easy and beneficial for further simulations. The suggested model is unique in that it picks and downloads a novel tagged dataset of genomic abnormalities from Kaggle. This dataset consists of 12,280 instances, 28 independent features, and one dependent feature (output class). Data were preprocessed in the early phases of this work, performing data normalization, replacing null or missing values applying different mean techniques, and splitting the dataset into two halves: training and testing.

The proposed model uses two machine learning techniques in the training phase: SVM and KNN for training on 70% of the dataset. The remaining 30% of the data is utilized for testing. As a consequence, based on the best accuracy, we chose the best-predicted model, which has been described in the simulation result section. Before we describe the simulation results it is appropriate to briefly describe the algorithms employed in this work.

### 3.1. Support Vector Machine

Support vector machine algorithm attempts to process the raw data onto a discrete feature space before generating an ideal interval hyperplane that can discriminate between positive and negative examples. We use a two-class SVM approach in this classification, and we create the training set using molecular sequences and interaction data, as reported in [27]. The positive training data includes all known illness genes, whereas the negative training data includes genes linked with new diseases and an additional 10% of genomic sequences.

The study [28] also uncovered EPI-related genes using a binary class SVM classifier. 69 binary characteristics of known PID and non-PID genes were combined to produce the classifier. The trained classifier identified 1,442 potential PID genes. In this work, a binary class SVM is trained on 29 functions and 70% of the dataset instances.

To show the characteristics of yi, linear combination variables *β*_i_ may be used to choose the vectors of the SVM hyperplane. A hyperplane relation is defined as [34, 35]:

(1) $$\begin{array}{c} \sum_{i}\beta_{i}k\left(y_{i},y\right)=m, \end{array}$$

where *k* is the kernel function *k*(*x*, *y*) and *m* is a constant.

Polynomial kernel function used for the training dataset is as follows [34–36]:

(2) $$\begin{array}{c} k\left(\overset{⟶}{y_{i}},\overset{⟶}{y_{j}}\right)={\left(\overset{⟶}{y_{i}}\cdot \overset{⟶}{y_{j}}\right)}^{d}, \end{array}$$

where *k* is the kernel function and *y* is the instance of features.

SVM classifier minimizes the variables by soft margins.

(3) $$\begin{array}{c} \left[\frac{1}{n}\sum_{i=1}^{n}\text{max}\left(0,1-m_{i}\left(z^{T}l_{i}-b\right)\right)\right]+ß{\left\|z\right\|}^{2}. \end{array}$$

The soft margins minimizing classifier is represented by equation (3) above, whereas the hard margins classifier is represented by *β*. Using a limited optimization problem, soft margin equation (3) can be rewritten as follows [37]:

(4) $$\begin{array}{c} \text{minimize}\frac{1}{n}\sum_{i=1}^{n}\zeta_{i}+ß{\left\|z\right\|}^{2}, \end{array}$$

where *i* = {1,…, *n*} and *ζi* is the smallest nonnegative number.

### 3.2. K-Nearest Neighbors

The KNN is a nonlinear predictive model developed in 1951 by Evelyn Fix and Joseph Hodges and later modified by Thomas Cover [28]. It is utilized in the segmentation and prediction of data. For both cases, the feed is a dataset containing the nearest *k* training sets. The outcome is determined by whether KNN is used for classifying or predicting. To improve prediction outcomes, the suggested model employed KNN for prediction and used a 70% training dataset to train the model based on features by varying the number of *k* folds. Statistical formation of KNN is given as [38]:

(5) $$\begin{array}{c} X|Y=x^{∼}Zr. \end{array}$$

In the KNN classifier, the *k*-nearest neighbors is given a weight of 1/*k*, while the remainder are given a weight of 0. The *j*^th^ nearest neighbor is assigned weight *f*_*nj*_ with [38].

(6) $$\begin{array}{c} w_{nj}=1. \end{array}$$

## 4. Dataset

We used the genome disorder dataset from Kaggle [39]. This dataset contains the medical histories of 12,280 people who have mitochondrial and multifactorial genetic inheritance disorders. There are 28 independent variables and one dependent variable in the genomic disorder dataset. In data preparation, the suggested model uses several missing value strategies to substitute null values.

## 5. Simulation Results and Discussion

SVM and KNN machine learning methods were used to train and test the proposed model. The classification accuracy, miss-classification rate, precision, sensitivity, and F1 score are used to evaluate these algorithms. The suggested model's initial stage involves preprocessing the data, replacing missing values, and dividing the data into two phases: training and testing. The suggested model is subsequently trained for the testing phase using SVM and K-NN machine learning methods. The simulation results from the proposed model are detailed below in terms of several prediction parameters. In the first phase, simulation results demonstrate confusion matrices of training and testing for both machine learning algorithms, and then the comparison of their parameters is presented in the second phase.

Table 2 shows the simulation parameters of the proposed model of SVM and KNN. It shows that the KNN model uses a total number of 5 neighbors with the exhaustive NS method, Minkowski distance between neighbors and standardize equals true. In parallel SVM uses a polynomial kernel function with auto kernel scale having 3 polynomial orders and standardize equals true.

The training confusion matrix of the SVM and K-NN algorithms can be seen in Table 3. The trained KNN model's confusion metric yields 6922, 657, 825, and 191 scores of true positive, true negative, false positive, and false negative, respectively. SVM received 6959, 1205, 277, 154 attributes of true positive, true negative, false positive, and false negative. As a result, the suggested model demonstrates that SVM obtains the greatest true positive rate when compared to the KNN model.

Table 4 depicts the prediction outcomes of both machine learning algorithms using the suggested model. The confusion metric for testing the K-NN model receives 3023, 115, 469, 77 attributes of true positive, true negative, false positive, and false negative, respectively, while the confusion metric for testing the SVM receives 2931, 262, 322, 169 attributes of true positive, true negative, false positive, and false negative.

The suggested SVM model Figure 2 gets the lowest mean squared error of 0.1089 after 24 epochs. It signifies that the suggested model's prediction results are accurate and efficient. Furthermore, this value has been improved by vary simulation hyper parameters, dataset with numerous numbers of iterations.

In Table 4 the accuracy, miss-classification rate, sensitivity, precision, and F1 score values are calculated by using the formulas mentioned below [37, 40–51].

(7) $$\begin{array}{c} \text{Accuracy}=\frac{\text{True Classified Instances}}{\text{Total Instances}},\\ \text{Miss}-\text{classification rate }=\frac{\text{False Classified Instances}}{\text{Total Instances}},\\ \text{Sensitivity}=\frac{\text{TP}}{\text{TP}+\text{FN}},\\ \text{Precision}=\frac{\text{TP}}{\text{TP}+\text{FP}},\\ F1\text{score}=\frac{2\text{TP}}{2\text{TP}+\text{FP}+FN}. \end{array}$$

The proposed model outcomes are analyzed using accuracy, miss-classification rate, precision, sensitivity, and F1-score analysis parameters.  Table 5 presents a comparison of all analytical parameters using the suggested machine learning model. The proposed K-NN model achieves accuracy, miss-classification rate, precision, sensitivity, and F1-score of 88.3 percent, 11.7 percent, 89.35 percent, 97.31 percent, and 93.15 percent, respectively. The proposed SVM-based model achieved 94.99 percent training accuracy, 5.01 percent, 96.17 percent, 97.83 percent, and 96.98 percent miss-classification Rate, precision, sensitivity, and F1-score, respectively. As a result, the suggested model demonstrates that SVM obtains the maximum training accuracy when compared to the KNN model. The suggested model outperforms state-of-the-art machine learning techniques in terms of prediction outcomes. The proposed KNN model achieves 85.1 percent, 14.9 percent, 86.56 percent, 97.51 percent, 91.7 percent prediction accuracy, miss-classification rate, precision, sensitivity, and F1-score, while the proposed SVM model achieves 86.6 percent, 13.4 percent, 90.10 percent, 94.54 percent, 92.26 percent prediction accuracy, miss-classification rate, precision, sensitivity, and F1-score. As a result, the suggested model demonstrates that SVM obtains the maximum prediction accuracy when compared to the K-NN model.  Table 6 shows the comparative analysis of previous studies with the proposed model and it shows Asif et al. [31] achieved 79% prediction accuracy empowered with RF and SVM used miRNA feature base dataset and having handcrafted features and imbalance data limitation, Alshamlan et al. [32] achieved 81% prediction accuracy empowered with GBC algorithm used SRBCT feature base dataset and having handcrafted features and imbalance gene sequence data limitation, KhaderKhader et al. [33] achieved 80.5% prediction accuracy empowered with BA and SVM used gene seq feature base dataset and having imbalance gene sequence limitation and on the other side the proposed model achieves 86.6% prediction accuracy empowered with SVM using genetic clinical feature based data and with IoMT technology. The proposed model achieves the best accuracy using the proposed model of SVM with the help of different simulation parameters which are far better than previously researched articles. So, it shows with the varying of simulation parameters models can get the best training and testing results.

## 6. Conclusion and Future Work

Smart machine learning plays a critical role in the early detection of genetic disorders. SVM and K-NN techniques were employed in this study to predict mitochondrial and multifactorial genetic inheritance disorders. The medical history of a patient provides significant information about a genetic problem, and this information is employed by the suggested model to forecast genetic inheritance disorders. SVM has the highest prediction accuracy of 86.6 percent, and it outperforms genetic sequence methods in terms of prediction performance. Patients and physicians will benefit from this research since it will allow them to predict gene abnormalities quickly and save lives. We also intend to develop this study in the future by using multiclass categorization of cancer, dementia, and diabetes, which will be extremely useful in the health care industry.

## Figures and Tables

**Figure 1:** IoMT-based proposed model for the prediction of genetic disorder.

**Figure 2:** Mean square error of support vector machine.

**Table 1:** Constraints and comparisons of previous studies.

Study	Model	Used dataset	Accuracy (%)	Constraint	IoMT
Asif et al. [31]	RF, SVM	miRNA (feature)	79	Handcrafted features, imbalance data	No
Alshamlan et al. [32]	GBC algorithm	SRBCT (feature)	81	Handcrafted features, imbalance classes, imbalance gene sequence	No
KhaderKhader et al. [33]	BA, SVM	Gene seq (feature)	80.5	Imbalance gene classes	No

**Table 2:** Simulation parameters of the proposed model of KNN and SVM.

Algorithm	Neighbors	NS method	Distance	Standardize

KNN	5	Exhaustive	Minkowski	True

SVM	Kernel function	Polynomial order	Kernel scale	Standardize
	Polynomial	3	Auto	True

**Table 3:** Training confusion metrics of the proposed model of KNN and SVM.

Total instances (8595)	1	2
SVM		
1	6922	191
2	825	657

KNN		
1	6959	154
2	277	1205

**Table 4:** Testing confusion metrics of the proposed model of KNN and SVM.

Total instances (3684)	1	2
SVM		
1	2931	169
2	322	262

KNN		
1	3023	77
2	469	115

**Table 5:** Performance of SVM and KNN models.

Instances (12280)	SVM		KNN	
	Training (%) (8596 instances)	Testing (%) (3684 instances)	Training (%) (8596 instances)	Testing (%) (3684 instances)
Accuracy	94.99	86.6	88.3	85.1
Miss-classification rate	5.01	13.4	11.7	14.9
Precision	96.17	90.10	89.35	86.56
Sensitivity	97.83	94.54	97.31	97.51
F1-score	96.98	92.26	93.15	91.7

**Table 6:** Comparative analysis with previous studies.

Study	Model	Dataset	Accuracy (%)	IoMT
Asif et al. [31]	RF, SVM	miRNA (feature)	79	No
Alshamlan et al. [32]	GBC algorithm	SRBCT (feature)	81	No
KhaderKhader et al. [33]	BA, SVM	Gene seq (feature)	80.5	No
**The proposed model**	**SVM, KNN**	**Gene clinical (feature)**	**86.6**	**Yes**

## Data Availability

The data used in this paper can be requested from the corresponding author upon request.
